The article "U-Net Modelling-Based Imaging MAP Score for Tl Stage Nephrectomy: An Exploratory Study" was retracted in 2023. Reasons: signs of a paper mill; suspected computer-generated content; unreliable results or conclusions; lack of ethics approval or compliance.

# U-Net Modelling-Based Imaging MAP Score for Tl Stage Nephrectomy: An Exploratory Study

**DOI:** 10.1155/2022/1084853

**Published:** 2022-01-05

**Authors:** Ruixue Sun, Ruiting Chang, Tianshu Yu, Dongxin Wang, Lijie Jiang

**Affiliations:** Imaging Department Hengshui People's Hospital, Hengshui 053000, China

## Abstract

We evaluate the stability of the clinical application of the MAP scoring system based on anatomical features of renal tumour images, explore the relevance of this scoring system to the choice of surgical procedure for patients with limited renal tumours, and investigate the effectiveness of automated segmentation and reconstruction 3D models of renal tumour images based on U-net for interpretative cognitive navigation during laparoscopy Tl stage radical renal tumour cancer surgery. A total of 5 000 kidney tumour images containing manual annotations were applied to the training set, and a stable and efficient full CNN algorithm model oriented to clinical needs was constructed to regionalism and multistructure and to finely automate segmentation of kidney tumour images, output modelling information in STL format, and apply a tablet computer to intraoperatively display the Tl stage kidney tumour model for cognitive navigation. Based on a training sample of MR images from 201 patients with stage Tl renal tumour cancer, an adaptation of the classical U-net allows individual segmentation of important structures such as renal tumours and 3D visualisation to visualise the structural relationships and the extent of tumour invasion at key surgical sites. The preoperative CT and clinical data of 225 patients with limited renal tumours treated surgically at our hospital from August 2011 to August 2012 were retrospectively analysed by three imaging physicians using the MAP scoring system for the total score and the variables *R* (maximum diameter), *E* (exogenous/endogenous), *N* (distance from the renal sinus), *A* (ventral/dorsal), *L* (relationship along the longitudinal axis of the kidney), and *h* (whether in contact with the renal hilum). The score for each variable (contact with the renal hilum) was statistically compared with each other for the three observers. Patients were divided into three groups according to the total score—low, medium, and high—and according to the surgical procedure—radical and partial resection. The correlation between the total score and the score of each variable and the choice of surgical procedure was analysed. The agreement rate of the total score and the score of each variable for all three observers was over 90% (*P* ≤ 0.001). The map scoring system based on the anatomical features of renal tumour imaging was well stabilized, and the scores were significantly correlated with the surgical approach.

The article "U-Net Modelling-Based Imaging MAP Score for Tl Stage Nephrectomy: An Exploratory Study" was retracted in 2023. Reasons: signs of a paper mill; suspected computer-generated content; unreliable results or conclusions; lack of ethics approval or compliance.

## 1. Introduction

The preoperative differentiation of benign and malignant renal tumours is very difficult, and most rare benign renal tumours cannot be distinguished from RCC on imaging, so according to the European Urological Association treatment guidelines, if the nature of the mass cannot be clearly determined, it should be treated in the same way as RCC [1]. With advances in surgical techniques, the primary method of resection for limited renal tumours has changed from RN to PN. Therefore, another important purpose of preoperative imaging in renal tumour patients is to provide a basis for the choice of surgical approach.

The choice of tumour resection and the prognosis depends largely on the anatomical complexity of the tumour, such as the size and location of the tumour. The most frequently analysed anatomical information about the tumour in imaging is generally sized, and there is a lack of description of signs, such as the location of the tumour in different parts of the renal parenchyma [2]. In the renal unit preserving approach, the overall relationship between the tumour and the kidney, such as the size of the tumour, its location within the renal parenchyma, its ventral and dorsal location, and whether it involves the renal hilum, needs to be clarified. The map scoring system was proposed in [3]. The MAP scoring system is a more comprehensive quantitative scoring method for assessing the anatomical complexity of renal tumours, which corresponds to the anatomical features of renal tumours with capital initials [4]. The variables are simple to set and relatively easy to measure [5].

The MAP scoring system is based on CT and MR images and uses axial and standard coronal reconstructions for observation, measurement, and scoring. As this scoring system is a quantitative data derived from the subjective, visual judgement of topographic images by the operator, it is subject to the operator's imaging experience and may vary between those with different experiences [6]. In this study, we evaluated the consistency of scoring by three different observers using the MAP scoring system independently and found that the consistency rate was above 90% for both total and individual scores, indicating that the scoring system is stable and reproducible [7]. This may be related to the professional background of the observer, who was a radiologist in this study, as opposed to a urologist in previous studies, and therefore may have had a more consistent understanding and measurement of the CT images.

In this study, we retrospectively analysed the preoperative anatomical imaging characteristics of 220 patients with renal tumours, scored them using the MAP scoring system, and investigated the correlation between the score and the surgical approach [8]. The results showed that MAP scores were significantly correlated with the choice of surgical procedure, with patients using the LPN procedure having significantly lower scores than those using the LRN procedure (*P* ≤ 0.001). The average total score for patients with the LPN procedure was 7.5, compared to 9.3 for patients with the LRN procedure. In the low group, 83.9% had the LPN procedure compared to 16.1% for the LRN procedure, while in the high group, 18.9% had the LPN procedure compared to 81.1% for the LRN procedure [9]. The results suggest that the lower the score, the lower the anatomical complexity of the renal tumour and the more the clinician tends to use the LPN procedure, while the higher the score, the higher the anatomical complexity of the renal tumour and the more the clinician tends to use the LRN procedure, which is in line with the foreign literature [10]. It is worth mentioning that in this group of patients, the preoperative surgeons did not decide on the surgical procedure based on this scoring system, but rather since the imaging features of the tumour are supplemented by operational experience, most of them successfully completed the operation according to the preoperative judgement, which may be related to the proficiency of the surgeons in our unit. This may be related to the proficiency of the surgeon in the unit. For those with less proficiency and experience, this assessment may be an important basis for the choice of procedure [1].

The article "U-Net Modelling-Based Imaging MAP Score for Tl Stage Nephrectomy: An Exploratory Study" was retracted in 2023. Reasons: signs of a paper mill; suspected computer-generated content; unreliable results or conclusions; lack of ethics approval or compliance.

When analysing the relationship between patient age, gender, affected side, and the individual items of the MAP scoring system and the choice of procedure, the items *R*, N, *L,* and *h* were all significantly correlated with the choice of procedure. The larger the tumour was, the closer it was to the renal sinus, the closer it was to the centre of the renal axis (nonrenal pole), the more difficult it was to partially resect, and the more radical surgery was required, and the older the patient was, the more radical surgery was preferred. There was no significant correlation between patient gender, affected side and score *E,* and the choice of procedure. Gao et al. [11] used the MAP scoring system to score 615 patients with renal tumours and evaluated the relationship between the scoring items and the choice of procedure and found that, in addition to *R*, N, *L,* and *h*, when the scoring item A (tumour located ventral or dorsal) was difficult to determine (marked as x), it was also significantly associated with the RN procedure.

The article "U-Net Modelling-Based Imaging MAP Score for Tl Stage Nephrectomy: An Exploratory Study" was retracted in 2023. Reasons: signs of a paper mill; suspected computer-generated content; unreliable results or conclusions; lack of ethics approval or compliance.

The weaknesses of this study are that it was a retrospective, single-centre study, which may have led to selective bias, particularly in terms of uneven surgeon proficiency, and that other clinical conditions of the patient's whole body were not analysed, which may have affected the interpretation of the results to some extent [12]. The decision to perform PN is an extremely complex process influenced by multiple factors, and the MAP scoring system is one of the comprehensive and reproducible preoperative imaging scoring systems currently used to evaluate tumour complexity, which can be used to assist in the screening of patients for proposed PN procedures [13].

## 2. Related Work

In recent years, with the popularity of deep learning research, CNNs have gained widespread attention. Stojmenovic and Lin [14] first proposed the use of multilayer CNN structures to discriminate handwritten characters in 1998, which was the cornerstone of CNNs for image processing. After decades of development, more and more scholars have applied CNNs to medical image data processing, and the segmentation and recognition of imaging organs are accomplished by “pretraining + structural fine-tuning” [15]. In [16], a three-dimensional CNN was applied to segment the vertebral body of MRI images. In [17], a deep 3D convolutional network was applied for multiscale feature fusion to segment the lesions of multiple sclerosis. Ayalew and Yamagishi [18] proposed a U-net for good cell wall structure segmentation of pathological compression slices of Hela (HeLa) cell suspension. Velkoska et al. [6] used a predefined ellipsoidal shape constraint in a Bayesian framework, which in turn segmented Tl stage renal tumours. Obajemu et al. [19] proposed a random forest-based algorithm to segment stage Tl renal tumours as a whole on CT images, with some results. Stage Tl renal tumours are an ellipsoidal dense organ with close density to muscle and fascia and low intertissue contrast, making segmentation difficult on conventional CT images. Katsura et al. [20] used U-net to combine CT and MR-T1WI data and combine the advantages of each to improve the segmentation accuracy of Dice (89. 59%) by 3%. In [21], based on a training set of 50 samples, a decomposition neural network was used to segment T2WI magnetic resonance images of stage Tl renal tumours, and a Dice similarity coefficient of more than 89.75% was achieved.

As the accuracy of imaging scans increases, the internal structures of the human body are being imaged with increasing clarity, and the segmentation and reconstruction of organs and fine structures are achieved through the remining image data [22]. Reference [11] applied 3D printing to assist cognitive navigation for physicians performing stage Tl renal tumour biopsies, increasing the positive puncture rate from 22.4% for systematic puncture to 46.2% for targeted puncture. In this study, the application of high-precision 3D reconstruction technology to assist the surgeon with cognitive navigation provided a good demonstration and understanding of an epiphytic tumour preoperatively and intraoperatively, and introspective observation and comparison in real time enabled complete resection of a difficult tumour, ensuring negative margins and surgical safety. Reference [23] applied display-based image overlay technology to achieve augmented reality navigation for partial hepatectomy. In the field of urology, [24] applied augmented reality technology to perform a difficult partial nephrectomy for a hilar tumour by manual alignment. Reference [25] was the first to demonstrate augmented reality simultaneous navigation for radical prostate cancer using TilePro multiscreen fusion technology at the American Urological Association annual meeting in 2013. In contrast, [26] reported an ultraprecise three-dimensional reconstruction (HA3D) augmented reality navigation technique using high-precision magnetic resonance, which effectively reduced the margin positivity rate in cases of extraterritorial invasion, while reducing the error between the 3D model and the whole pathology section to the 3 mm level. This study integrates the techniques and efforts of image segmentation, recognition, alignment, 3D reconstruction, neural network design, and pathology proofreading, but the realistic deficiencies faced are reflected in all aspects, such as segmentation.

The article "U-Net Modelling-Based Imaging MAP Score for Tl Stage Nephrectomy: An Exploratory Study" was retracted in 2023. Reasons: signs of a paper mill; suspected computer-generated content; unreliable results or conclusions; lack of ethics approval or compliance.

## 3. Model Proposed

### 3.1. Image Acquisition and Parameters

A multiparametric MRI was performed prior to stage Tl renal tumour puncture using a Siemens 3.0 T MRI scanners with an abdominal phased array coil to receive the signal. Diffusion imaging axial scans were performed using a single excitation planar echo (EPI) sequence, and the magnetic resonance scanner automatically calculated ADC images, exported 1 mm thick thin DICOM data, and applied RadiAnt DICOM Viewer V4.6.5 to obscure basic patient information for post-automated segmentation [27–30].

### 3.2. Structural Design of the U-Net

Based on the classical U-net proposed by reference [20] in 2015, a simple structured U-net with an excellent performance was constructed by adapting it. The original MRI image of 320 × 320 pixels is first centrally cropped into a 256 × 256-pixel image input image tile. On the left side of the network is the contradiction, which is a series of degraded acquisition operations consisting of Max pooling. The compression path consists of four blocks, resulting in a feature map of 16 × 16 pixels in size. The right-hand side of the network is the expansive path, which also consists of 4 blocks, each of which is started by deconvolution, and then merging it with the feature map of the symmetric compressed path on the left-hand side [31,32].

The article "U-Net Modelling-Based Imaging MAP Score for Tl Stage Nephrectomy: An Exploratory Study" was retracted in 2023. Reasons: signs of a paper mill; suspected computer-generated content; unreliable results or conclusions; lack of ethics approval or compliance.

The feature map in the compressed path is slightly larger and is trimmed for stitching. The convolution operation for the extended path is still an effective convolution operation, resulting in a feature map size of 256 × 256 pixels.  Figure 1 is architecture of the modified U-net.

In order to give the network the ability to separate the boundaries, we designed the loss function with boundary weights:

(1) $$\begin{array}{c} E=\sum_{X\in \Omega }\omega \left(X\right)\log\left(p_{\ell \left(X\right)}\left(X\right)\right). \end{array}$$

Here, *p*_*ℓ*(*X*)_(*X*) is the SoftMax loss function, *ℓ* : Ω⟶(1,…, *k*) is the label value of the pixel point, and *ω* : Ω ∈ *R* is the weight of the pixel point, in order to give higher weights to the pixels close to the boundary points in the image:

(2) $$\begin{array}{c} \omega \left(X\right)=\sqrt{\omega_{c}\left(X\right)}+\;\omega_{0}\cdot \;\exp\left(-\frac{{\left(d_{1}\left(X\right)+d_{2}\left(X\right)\right)}^{2}}{2\sigma^{2}}\right). \end{array}$$

Here, *ω*_*c*_ : Ω ∈ *R* is the weighting of the proportion of balanced categories, *d*_1_ : Ω ∈ *R* is the distance from the background pixel to its nearest segmentation label, and *d*_2_ : Ω ∈ *R* is the distance from the background pixel to its second closest segmentation label. *ω*_0_ and *σ* are constant values in the experiment. Conversely, *ω*_0_=10,  *σ* ≈ 5, and the above operation is done again from the segmented label pixel point to its nearest and second closest background pixel point. This gives a weight to the ground truth, as shown in the C diagram in Figure 2, where a brighter color indicates a higher weight and a higher penalty if the network makes an incorrect decision at the corresponding pixel, thus substantially improving the effectiveness of edge segmentation.

In this study, the Tl kidney tumour and its surrounding structures (e.g., bilateral seminal vesicle glands and rectum) were segmented independently in order to meet the need for refined surgical navigation [33–35]. In contrast to the conventional classical U-net, the “conv 3 × 3, ReLU” step was optimised to “conv 3 × 3, batch normalization, ReLU” to speed up the convergence of the model and to alleviate some of the problems associated with the deeper model. In addition, we apply a square root to *ω*_*c*_(*X*), so that the network learns with focus without overlooking the background. At the same time, both sides of the segmented category contours in ground truth are strengthened with weights, and by adjusting the degree of strengthening, the inner side is stronger, so that the training results tend to favour larger contours, which is effective in practical navigation applications. The training results thus tend to favour larger contours, which serve to effectively reduce cut edge positivity in practical navigation applications. The training set used in this study contains about 201 cases (24–30 images per case, about 5,000 images in total), and any form of data augmentation has been discarded to ensure the real reliability of the network. All training was based on the original image segmentation. Figure 2 shows example of U-net segmentation of a stage Tl renal tumour and adjacent structures.

The article "U-Net Modelling-Based Imaging MAP Score for Tl Stage Nephrectomy: An Exploratory Study" was retracted in 2023. Reasons: signs of a paper mill; suspected computer-generated content; unreliable results or conclusions; lack of ethics approval or compliance.

In a test set application containing 98 Tl stage renal tumour cancer multiparametric MRI images, we used a modified U-net for automated segmentation without any preprocessing and calculated warping error, Randerror, and pixel error. The network achieved a warping error of 0.000 340 and a Randerror index of 0.036 0, with a Dice similarity coefficient of 90%, compared with manual segmentation and the application of previously reported deconvolutional networks complexes.  Table 1 is comparison of U-net performance with other segmentation effects.

### 3.3. Cognitive Navigation

The STL data are imported into an android tablet and viewed using the STL Viewer V2.0. The operator is asked to learn the structure of the 3D model of a stage Tl kidney tumour in conjunction with MRI before surgery. During the operation, the assistant manipulates the 3D model in real time according to the surgical view. The 3D model is displayed on the table and the surgeon performs the separation and manipulation of the fine structures [13].

## 4. Case Studies

Preoperative CT (plain + enhanced) data and clinical data of patients undergoing surgical resection (RN or PN) for renal tumour in our hospital from August 2011 to August 2012 were collected. The exclusion criteria were (i) the presence of venous thrombosis, invasion of adjacent structures or metastases as determined by CT; (ii) patients with absolute indications for PN, such as isolated kidney or contralateral renal dysfunction, bilateral multiple renal tumours; and (iii) unilateral multiple tumours. The MAP scoring system and criteria are based on the following six aspects: radius (R), epiphytic (E), distance from the renal sinus and collecting system (N), whether the tumour is located ventral to the kidney (A), location along the longitudinal axis of the kidney (L), whether there is a relationship with the blood vessels of the kidney (hilar, h), and whether there is contact with the vessels of the renal hilum. The total score of the MAP scoring system was divided into three groups of low (4–6), medium (7–9), and high (10–12) score, as described in [15]. The images were analysed and scored by radiologists, one junior resident, one senior resident, and one attending physician individually, using an online tool to score each item independently. Three physicians had studied the MAP scoring system and mastered the scoring criteria before scoring and were unaware of the procedure and postoperative pathology the patient had undergone at the time of scoring. The images included both axial and standard coronal reconstructions, and the image of the clearest tumour border was selected for observation, measurement, and scoring (generally enhanced scans were selected).

The article "U-Net Modelling-Based Imaging MAP Score for Tl Stage Nephrectomy: An Exploratory Study" was retracted in 2023. Reasons: signs of a paper mill; suspected computer-generated content; unreliable results or conclusions; lack of ethics approval or compliance.

### 4.1. Surgical Selection and Execution of Renal Tumour Resection

There are four types of nephrectomies: laparoscopy partial nephrectomy (LPN), open partial nephrectomy (OPN), open radical nephrectomy (ORN), and laparoscopy radical nephrectomy (LRN). The proposed and actual preoperative procedures are documented in the medical record, and if not, the reasons for the change of procedure are recorded.

### 4.2. Results

A total of 225 patients were included in this study, with an average age of 51.9 ± 11.6 years (24 to 83 years), of whom 149 were males and 76 were females. The average age of patients was 51.9 ± 11.6 years (24–83 years), with 149 males and 76 females. All patients had a single tumour in the kidney with a mean size of 4.6 ± 2.4 cm (1.2–20.0 cm). Preoperative PN was proposed in 103 patients (102 for LPN and 1 for OPN) and RN in 122 patients (118 for LRN and 4 for ORN). Three patients were converted from LPN to LRN. The reason for the conversion was a large amount of interpretative bleeding due to changes in the renal artery. Postoperative pathology confirmed that the tumours were predominantly renal cell carcinoma in 180 cases (80%), benign tumours in 40 cases (17.8%), and a few rare tumours.

The concordance rates and Kendall's Harmony coefficients for the MAP score of the three different observers are shown in Table 2. Among the three observers, the concordance rate for the total score was 97.1%. The highest concordance rate for the six items in the rating system was *h* (98.6%), followed by *R* (96.4%), A (95.6%), and N (94.3%), and the lowest concordance rate was *L* (90.7%), followed by *E* (93.7%). The *P* value for all items including the total score was <0.05, suggesting that the difference was statistically significant. Table 2 presents consistency of MAP scores.

The article "U-Net Modelling-Based Imaging MAP Score for Tl Stage Nephrectomy: An Exploratory Study" was retracted in 2023. Reasons: signs of a paper mill; suspected computer-generated content; unreliable results or conclusions; lack of ethics approval or compliance.

The numbers of cases with low (4–6), medium (7–9), and high (10–12) score were 31 (13.8%), 115 (51.1%), and 79 (35.1%), respectively. Five of the cases had open surgery (ORN1 and OPN4) and were not included in the statistical analysis due to the small number of cases. The surgical procedures were divided into LRN (121 cases) and LPN (99 cases). In the low, medium, and high groups, there was a decreasing trend of 83.9%, 51.3%, and 18.9% for the LPN procedure, respectively; on the other hand, there was an increasing trend for the LRN procedure. The mean total score for patients with the LPN procedure was 7.5, while the mean total score for patients with the LRN procedure was 9.3. The relationship between the total score and the choice of procedure was analysed using the rank sum test and the difference was significant (*P* ≤ 0.001), with patients with the LPN procedure having a lower total score than those with the LRN procedure.  Table 3 displays total MAP score and implementation of the procedure.

Multiple logistic regression analysis was used to analyse the relationship between patient gender, age, affected side, and each score item *R*, *E*, *N*, *A*, *L,* and *h,* and the choice of surgical procedure. The items associated with the choice of procedure were *R*, *N*, *L,* and *h* (*P* < 0.05). The higher the *R*, *N*, and *L* scores were, the more the tumour was in contact with the renal vessels (h) and the more the LRN procedure was favoured, and conversely the LPN procedure was favoured (*P* values 0.000, 0.034, 0.034 and 0.012 respectively). In addition, the younger the age, the greater the preference for LPN (*P* = 0.019). There was no significant correlation between gender, affected side and scores *E* (epiphytic or not) and A (ventral or dorsal) and the choice of procedure (*P* > 0.05).  Table 4 shows analysis of factors influencing the choice of procedure.

## 5. Analysis of Experimental Results

The tumour visualisation is presented in the following. A male patient, 73 years old, was found to have total PSA (T-PSA) 30.0 ng/m *L* and free PSA (F-PSA) 3.87 ng/m *L*, F/T = 0.13; magnetic resonance findings suggested that the tumour was predominantly ventral, with the basal tumour protruding superiorly and the local. The tumour was mainly located on the ventral side, with the basal tumour protruding upwards and the envelope blurred. The operation was completed successfully, with a duration of 165 min and a blood loss of 50 m L. The bilateral neurovascular bundle was not preserved during the operation due to severe adhesions, and the postoperative urinary catheter was left in place and removed after 2 weeks. The total length of stay was 7 d. The postoperative pathology showed a stage Tl renal tumour with alveolar carcinoma, mainly in the ventral basal part, involving the left and right lobes, with the basal tumour convex to the upper left. The whole pathological section was highly compatible with the 3D reconstruction model.  Figure 3 shows magnetic resonance T2WI image of the patient's stage Tl renal tumour.

The article "U-Net Modelling-Based Imaging MAP Score for Tl Stage Nephrectomy: An Exploratory Study" was retracted in 2023. Reasons: signs of a paper mill; suspected computer-generated content; unreliable results or conclusions; lack of ethics approval or compliance.

In the case of renal (2 + 1 suture, personalized subgroup 5), the renal tumour is removed, the broken vessels and collecting system of the renal wound are sutured, the renal artery is opened, and the renal wound is carefully closed with successive sutures after rapid and widely spaced suturing of the renal wound margin.  Figure 4 is standard nonblocking technology.  Figure 5 is preexisting sutures without blocking technique.  Figure 6 is preoperative DSA superselective embolization without blocking technique.  Figure 7 is early sequential open blood flow method.  Figure 8 is the “2 + 1” suture method.

In 97 patients with renal tumours, a personalized “shortening of thermal ischaemia” protocol was designed, of which 83 (85.6%) underwent personalized partial nephrectomy according to the personalized protocol (personalized group).

In the personalized subgroup 1 (standard unobstructed partial nephrectomy), 17 patients (17/20, 85.0%) completed the operation, while 3 patients were converted to renal artery block (2 + 1 suture) due to high interpretative bleeding; in the personalized subgroup 2 (reserved suture unobstructed technique), 15 patients (15.0%) completed the operation.

In personalized subgroup 2 (preselected suture without blocking technique), 15 patients (15/19, 78.9%) completed the procedure and 4 were converted to 2 + 1 sutures, of which 2 had completely endogenous tumours and 2 had excessive interpretative bleeding; in personalized subgroup 3 (preoperative DSA superselective immobilization without blocking technique), 12 patients (12/17, 70.6%) completed the procedure and 5 were converted to 2 + 1 sutures, of which 3 had preoperative interventions that failed to precisely locate the superselective tumour supplying the tumour. In the personalized subgroup 4 (early sequential opening), 18 patients (18/20, 90%) completed the procedure and 2 were converted to 2 + 1 sutures, of which 2 had severe adhesions in the hilum, resulting in unclear anatomical levels of the renal artery branches. In subgroup 5 (“2 + 1 suture”), all 21 patients enrolled had a personalized design.

There was no statistically significant difference in the preoperative renal function assessment between the personalized group and the conventional group (*P* = 0.33). On postoperative day 2, there was no statistically significant difference in the loss of renal function between the personalized and conventional groups. As the postoperative period progressed, the recovery of renal function was significantly better in the personalized group than in the conventional group. At 6 and 12 months postoperatively, the personalized group showed a statistically significant difference in the recovery of renal function (6 months *P* = 0.04, 12 months *P* ≤ 0.001). In order to further clarify the differences between the subgroups in the individualized group, we compared the tumour diameter, R.E.N.A.L score, operative time, thermal ischaemia time, interpretative bleeding, preoperative, and postoperative renal function at 12 months between the groups.

The article "U-Net Modelling-Based Imaging MAP Score for Tl Stage Nephrectomy: An Exploratory Study" was retracted in 2023. Reasons: signs of a paper mill; suspected computer-generated content; unreliable results or conclusions; lack of ethics approval or compliance.

## 6. Conclusions

This paper presents the effectiveness of interpretative cognitive navigation for laparoscopy stage Tl renal tumour cancer radical surgery based on an automated 3D model of renal tumour image segmentation and reconstruction built by U-net. A stable and efficient full CNN algorithm model oriented to clinical requirements was constructed for regionalism, multistructural, and fine-grained automated segmentation of renal tumour images. Based on a training sample of magnetic resonance images from 201 patients with stage Tl renal tumour cancer, a separate segmentation of important structures, such as renal tumours, could be achieved through adaptive improvement on the basis of the classical U-net, and 3D visualisation was performed intuitively. The structural relationships and the extent of tumour invasion at key surgical sites are visualized.

## Figures and Tables

**Figure 1:** Architecture of the modified U-net.

**Figure 2:** Example of U-net segmentation of a stage Tl renal tumour and adjacent structures.

**Figure 3:** Magnetic resonance T2WI image of the patient's stage Tl renal tumour.

**Figure 4:** Standard nonblocking technology.

**Figure 5:** Preexisting sutures without blocking technique.

**Figure 6:** Preoperative DSA superselective embolization without blocking technique.

**Figure 7:** Early sequential open blood flow method.

**Figure 8:** The “2 + 1” suture method.

**Table 1:** Comparison of U-net performance with other segmentation effects.

Croup name	Warping error	Rand error	Pixel error
Human values	0.000004	0.0019	0.0009
Zhan	0.000410	0.0367	0.0688
U-net	0.000340	0.0360	0.0596

**Table 2:** Consistency of MAP scores.

Component	Frequency of concordance (%)	Kendall, *s* coefficient of concordance	*P* value
R	96.4	0.980	≤0.001
E	93.7	0.963	≤0.001
N	94.3	0.933	≤0.001
A	95.6	0.972	≤0.001
L	90.7	0.938	≤0.001
H	98.6	0.985	≤0.001
Sum	97.1	0.990	≤0.001

**Table 3:** Total MAP score and implementation of the procedure.

Surgical options	4–6	7–9	10–12
LRN	5(16.1)	56(48.7)	60(81.1)
LPN	26(83.9)	59(51.3)	14(18.9)
Total	31(100)	115(100)	74(100)

The article "U-Net Modelling-Based Imaging MAP Score for Tl Stage Nephrectomy: An Exploratory Study" was retracted in 2023. Reasons: signs of a paper mill; suspected computer-generated content; unreliable results or conclusions; lack of ethics approval or compliance.

**Table 4:** Analysis of factors influencing the choice of procedure.

Variants	LRN	LPN	*P* value	B
Gender	82/39	65/34	0.561	−0.221
Age/years	53.6 ± 11.1	49.4 ± 11.7	0.019	0.038
Laterality	55/66	48/51	0.543	0.220
R1/2/3	29/74/18	78/18/3	0.000	1.807
E1/2/3	44/41/36	40/31/28	0.280	0.251
N1/2/3	4/3/114	20/12/67	0.034	0.686
L1/2/3	21/11/89	51/4/44	0.034	0.414
H-/h	85/36	98/1	0.012	2.789

## Data Availability

The simulation experiment data used to support the findings of this study are available from the corresponding author upon request.
